# A Study on the Relationship between Painter's Psychology and Anime Creation Style Based on a Deep Neural Network

**DOI:** 10.1155/2022/7761191

**Published:** 2022-07-05

**Authors:** Pei Wu, Sijie Chen

**Affiliations:** Hunan Normal University, College of Engineering and Design, Changsha, Hunan 410000, China

## Abstract

We conduct an in-depth study on the model construction of deep neural networks and design a model of painter's psychology and anime creation style to realize the study of the relationship between painter's psychology and anime creation style based on deep neural networks. This paper proposes an animation creation psychology classification algorithm that integrates human cognitive deep network structure optimization. The algorithm analyzes the connection between different convolutional layer features and animation characteristics through animation creation style CNN feature visualization. It interactively uses the knowledge of animation creation psychology expression techniques to optimize the network structure. This paper proposes a scene animation network based on spectral difference perception style. By analyzing the characteristics and differences in the spectrum between realistic and anime domain images, the generator is guided to learn the mapping relationships better to fit the style distribution of anime domain images. This paper uses a fully convolutional structure; the network is more lightweight and supports image inputs of arbitrary size, which can keep the semantic system of the background unchanged while highly deforming the five facial features, moving toward the goal of human-scene fusion for the animation task.

## 1. Introduction

From a theoretical point of view, the study of animation of images and videos is a study of computer vision. While improving the quality and stability of image translation tasks, we explore the space and ability of machines in “imitation and creation.” In terms of application value, the combination of realistic scene animation, which retains the semantic information and content characteristics of the natural world and has the style characteristics and artistry of the secondary genre, has a wide range of scenarios in current social media and short video applications, such as user avatars and fast video creation [1]. The use of machine learning to integrate realistic scenes with the secondary genre allows everyone to become a creator. To a certain extent, the development of anime and manga can even directly participate in creating film and television, providing new categories for film and television resources [2]. In recent years, machine learning methods based on deep neural networks have succeeded in computer vision, and advanced vision tasks such as image-to-image translation work have attracted many scholars. Using artificial intelligence to extract information from an image's external appearance and underlying features can access more than human eye perception and practical brain learning, making computer vision a further step in imitation and autonomous creativity [3]. This allows greater possibilities and room for play in the translation of images and lays the technical foundation for the large-scale implementation of AI-assisted image creation.

With the emergence of large-scale, high-quality datasets (e.g., Image Net), deep learning techniques have achieved breakthrough image cognitive layer recognition results [4]. Compared with artificially designed features, the unique multilayer structure of deep learning enables it to learn in-depth features that gradually transition from pervasive underlying visual elements (e.g., edges, textures, etc.) to higher-level semantic representations (torso, head, etc.) and the deeper the level, the more expressive it is. The hierarchical nature of depth features provides a proven way to bridge the semantic gap and achieve a cognitive understanding of emotions [5]. Therefore, many researchers have also applied deep learning to natural images for emotion recognition. However, unlike realistic images, the annotation of abstract image datasets requires hiring high-level experts and designing specialized annotation tools, which results in the available datasets being insufficient to train a deep, deep learning model [6]. The scarcity of annotation can lead to serious overfitting problems of deep learning models, and how to solve the overfitting problem of deep learning for learning tasks with small sample datasets has become a research hotspot in the field of computer vision.

Transfer learning is a significant research problem in machine learning. The goal is to apply knowledge or patterns learned in one domain or task to a different but related field or situation [7]. Transfer learning attempts to achieve the human ability to learn by analogy, such as applying skills gained from learning to ride a bicycle to learning to ride a motorcycle and knowledge gained from learning photography to painting. The main idea is to use the richly labeled source domain to improve the sparsely labeled target domain [8]. Transfer learning techniques have also been widely used in deep learning. Fine-tune pretrained deep networks on Image Net or Places datasets are a common strategy to learn specific in-depth features and alleviate the problem of small dataset samples. However, existing migration learning methods still have many issues, such as the undermatching problem caused by the difference in probability distribution between the source and target domains and the harmful migration problem where the source domain task hurts the target domain task.

## 2. Related Works

Image animation belongs to a kind of stylization, and image stylization can be understood as the process of image rerendering. In graphics, image stylization rendering techniques can theoretically be divided into three categories: methods based on stroke rendering, image analogy methods, and image filtering methods [9]. The earliest stylization almost always rerendered the original image according to artificially defined rules. There are ColorMatrix-based methods to perform independent transformations on individual pixels, capable of adjusting the brightness, contrast, saturation, hue, etc.; there are convolution-based methods that use different convolution kernels to perform convolution operations on the image, capable of edge enhancement, embossing there are also methods based on affine transformation matrix, which can rotate, scale, and tilt the image globally or locally [10]. The images are stylized using different processing techniques blended to achieve a specific style. Most of these processing techniques can be called filters, and their drawback is that the generated images are less realistic and have a more solidified style [11].

In 2018, Carto〇nGAN was proposed for the anime stylization problem. The model introduced a content loss function that controls the semantic information of the generated images by imposing this loss function separately for pretraining, so there is no need to use a loop structure [12]. In addition, for anime images with precise edges, an edge-boosting adversarial loss function is designed to blur the boundaries of anime images, allowing the discriminator to recognize such erroneous examples and thus controlling the model to generate ideas with transparent edges [13]. It utilizes unpaired training data and a one-way GAN structure to realize the conversion from realistic to anime scenes. In 2019, Ani Megan was improved based on Cartoon GAN; three loss functions enhance anime vision: grayscale antagonistic loss, grayscale style loss, and color reconstruction loss, which better maintains the color distribution of the original image and generates quality better anime images [14]. The limitation of these methods is that they can only animate stylized backgrounds such as buildings and landscapes and cannot highly animate abstraction of the five features of a human face [15]. There is a significant difference between anime faces and real faces, and it is not only the strokes, textures, and color styles but also the semantic and contour features of the five senses that need to be transformed. U-GAT-IT follows the structure of a recurrent consistent adversarial network, introduces an attention module to help the model find the regions that need to be highly charged, and proposes A novel AdaptiveLayer-InstanceNormalization (AdaLIN) method is proposed to control the amount of shape and texture variation and enhance the model robustness [16]. The study successfully achieves the conversion between natural human face and anime face. The shortcomings are that the model uses fully connected layers, which makes the image pixels compressed, resulting in blurred background and loss of some details, and the model is too large and not easy to train and deploy [17].

The latest deep learning-based methods are initially for oil painting art style migration tasks, do not capture the texture and color characteristics unique to cartoon images well, and are not satisfactory for cartoon rendering directly; the main drawback of such methods is that the generated results contain many artificial traces (Artifacts) [18]. These methods cannot make a good trade-off between global image style conversion and local image semantic content details maintenance, so the semantic details in the image are often lost. In 2018, Ekawardhani et al. proposed an adversarial generative network (Cartoon GAN) for cartoon-style migration based on adversarial generative networks, which can achieve cartoon-style rendering of realistic images [19]. Still, the model trained by this method can only handle a single cartoon substyle (e.g., Hayao Miyazaki's style and Makoto Shinkai's style are different cartoon substyle), and this method cannot take high-resolution images [20]. Bau et al. proposed an anime-style rendering network for selfie face images, using generative adversarial network techniques combined with spatial attention mechanisms so that the network learns the mapping relationship from natural face images to corresponding cartoon face images [21]. This approach requires pairs of face images and related cartoon face images as training data.

## 3. Model Construction of Deep Neural Networks

A convolutional neural network is the most widely used among various deep neural networks. It has achieved better results in many problems of machine vision and its successful applications in natural language processing, computer graphics, and other fields. CNN (convolutional neural network) is a variant of a traditional neural network; CNN introduces convolution and pooling based on a conventional neural network. Compared with a conventional neural network, CNN is more suitable for use in images; convolution corresponds to the local features of the image, and pooling makes the feature obtained by convolution spatially invariant. A convolutional neural network that is quite efficient for handwritten character recognition is proposed, the originator of many current convolutional neural networks [22]. As shown in Figure 1, the Le Net network consists entirely of a convolutional layer and a fully connected layer. After inputting handwritten characters into the network, the features are extracted by convolution, and the results are finally output as ten different classes.

### 3.1. Convolutional Layer

The convolutional layer is the essential operation in the convolutional neural network. Its core is to obtain the local information of the image by the convolutional kernel of a specific size acting on the local image area. A convolutional layer contains multiple convolutional kernels, and a single convolutional kernel convolves all the input feature maps to obtain the output feature map set. Hence, the number of output feature maps is the same as that of convolutional kernels. Suppose *A*^(*l*)^ is the output of the *l* convolutional layer of the convolutional neural network (*A*^(*o*)^ the web's input image); then, the *i*(*l* < *i* < *m*^(*l*)^) feature map can be expressed as follows:

(1) $$\begin{array}{c} A_{i}^{l}=\sum_{j=1}^{m^{l}}A_{j}^{l}⊗b_{i}^{l}. \end{array}$$

The weights of the convolutional layers can be generated by random initialization or by migrating the consequences of the convolutional layers of the same network structure trained on a large-scale dataset. Each element of the same feature map is obtained by convolving the input feature map with the same convolutional kernel, a shared weights feature. The shared weights feature means that the convolution kernel has fixed weights when traversing all input feature maps; i.e., all elements in the entire output feature map “share” the same convolution kernel. Thus, the convolution kernel can also be understood as a filter template. In addition to weight sharing, in each convolution operation, each convolution kernel acts only on a local region of the input image or feature, rather than directly on the whole image or part, a feature called locally connected [23]. This practice is derived from the biological neural system theory where neurons in the human brain only receive output from upper neurons within a particular spatial range. Images are a structured data source, where neighboring pixels may be closely related to each other, while pixels farther apart may be disconnected from each other. Therefore, each neuron only needs to take the local elements around the neuron as input and not the entire image pixel points as input. These two features, weight sharing and regional connectivity, improve the performance of convolutional neural networks and significantly reduce the number of parameters of the network.

### 3.2. Activation Layer

After the convolution layer, the output data is generally fed into the activation function, also known as nonlinearity mapping. The activation function adds nonlinear operations to the output obtained from linear operations to get a more robust feature transformation capability. Therefore, deep neural networks can theoretically approximate models of arbitrary functions, including complex nonlinear models. The Sigmoid function, also known as the S-shaped function, maps the input domain between 0 and 1. Assuming that the input data is *x*, the activation function (*x*) is defined.

(2) $$\begin{array}{c} \text{Sigmoid}\left(x\right)=\sum \frac{1}{\sqrt{e^{x}-1}}. \end{array}$$

The Sigmoid function can well model the properties of biological neurons: when the total amount of input signal received by a neuron breaks through a certain threshold, the neuron is activated and is excited; otherwise, it is in an inhibited state. In addition, the derivative of the Sigmoid function is *σ*′=*σ∗*(1 − *σ*); i.e., its result can be expressed in terms of itself, which is convenient for the calculation of the backpropagation method. However, the closer the Sigmoid function is to the origin, the larger the slope of the curve is, and the farther it is from the source, the closer the pitch is to 0. Therefore, if the initial weight of the network is too large, the neurons will quickly reach the saturation state, which will make the gradient of the output tend to 0. This will make the Tanh function: Tanh function, also known as the hyperbolic tangent function, is a deformation of the Sigmoid function, whose function curve is like the Sigmoid function; the difference is that its output domain is between −1 and 1. Its formula is defined as follows:

(3) $$\begin{array}{c} \sigma_{\left(x\right)}=2\text{Sigmoid}\left(2x\right)-\frac{\sqrt{e^{x}+e^{-x}}}{e^{x}-1}. \end{array}$$

### 3.3. Pooling Layer

After the stream's data has passed through the convolution and activation layers, a pooling layer is sometimes added for processing. As shown in Figure 2, the purpose of the pooling layer in the left half is to extract the main features and reduce the amount of data by subsampling the input data. Standard pooling methods are Max-pooling, Mean-pooling, and Stochastic-pooling. The right half shows the Max-pooling operation on a single feature graph: a 2 × 2 window is used to traverse the entire input feature graph from doing to right, top to bottom, in a particular step, and all the data in the window are taken as the maximum value and then used as the output. Averaging pooling means averaging all the data within the local window, while random pooling involves randomly selecting features in each pooling region based on a polynomial distribution. The pooling layer not only plays the role of downscaling and feature aggregation but also has specific translation, rotation, and scale invariance, which makes the convolutional neural network robust to image-related tasks and demonstrates its importance in the field of computer vision.

### 3.4. Fully Connected Layers

After several layers of convolution, activation, and pooling, the features of the input image are abstracted from the original pixel values to high-level semantic features, which are then mapped to the label space through the fully connected (FC) layers. Each neuron in the fully connected layers is connected two by two to each neuron in the previous layer, so all neurons influence the output of each neuron in the last layer. The fully connected layer is usually placed after the previous convolution and pooling operation in convolutional neural networks. Its primary role is to compress the feature map tensor into a feature vector for easy input into the classifier [24]. In addition, the fully connected layer can also be used as a classifier. The previous convolutional, activation, and pooling layers abstract the input data layer by layer to extract the high-level semantic features. The fully connected layer maps the high-level semantic features into the label space, thus achieving the classification. However, since each neuron in the fully connected layer is related to all neurons in the previous layer, it leads to an excessive number of its parameters, which increases the computational cost and causes overfitting problems. Therefore, some mainstream neural network models such as Google Net and Res Nel use the global average pooling (GAP) layer instead of the fully connected layer, which reduces the parameters of the network by nearly 80% and effectively speeds up the training of the model. Google Net focuses on deepening the network structure while introducing a new fundamental system, the Inception module, to increase the width of the network. The residual module is presented. A convolutional neural network is a multilayer neural network consisting of a stack of convolutional layers, activation layers, pooling layers, and fully connected layers. The convolutional layer is characterized by weight sharing and sparse connectivity, which can effectively extract structured features and reduce computational effort; the activation layer can perform nonlinear operations; the pooling layer can compress features and make feature representation more robust, and the fully connected layer can map high-level semantic features to the labeled space for classification [25]. There are also many differences in the feature patterns extracted by the different layers of the convolutional neural network. The closer the input layer is to the underlying visual features (e.g., edges, textures, etc.), the closer the classifier is to the features. The more abstract and discriminative semantic information is extracted. A simple linear classifier can be used for classification in the end.

## 4. Painter Psychology and Animation Creation Style Model Design

A series of works studying animation, such as Cartoon GAN and Ani Megan, summarize the stylistic features of anime images, such as having clear borders, sparse color blocks, high saturation, and manually design the relevant loss functions to make the mapping relationships gradually approach these features during the iterative process, so that the generated images can have the characteristics of anime images in visual senses. However, these algorithms are based on the extraction of different features and the matching of the weights between the elements, which are only part of the external representation of the anime image and do not represent the complete style of the painting, resulting in the gap between the style of the generated image and the style of the anime image in the target domain. In addition, the ideas generated by these algorithms will have unstable color changes or overall color shifts, which makes the realism and reproduction of the generated images poor. The loss of image details also makes the overall quality of the photos not high enough. Therefore, this section proposes a loss function based on spectral features, which abstracts the potential style representation in the image domain from the perspective of the frequency domain, and combines with the boundary loss function and color block loss function to provide a more comprehensive perception of the style of anime images for more adaptive anime conversion of ideas. The generated images are of higher quality and better in realism and color reproduction than the above network models.

Under the condition that there are paired data sets for training, the network can better learn the mapping relationship between domains through conditional constraints such as color distribution and texture details. The discriminator can have more information to discriminate the authenticity of the input images. For anime studies lacking paired training datasets, it is not difficult to judge the unknown potential distribution from two photos with entirely different semantic information [26]. According to the summary of the characteristics of anime domain images, it can be understood that the discriminator network needs to judge the attributes of color richness, edge sharpening, and color block sparsity in a set of images. Another comparison of the same semantic map with AnimeGAN for anime transformation between the existing domain and anime domain spectrum is shown in Figure 3. It can be observed that there are indeed apparent differences between the two types of images. The actual domain images are generally brighter and scattered, with less regularity (linear or textured).

In contrast, the animation domain images are usually more distinct in light and dark areas, with more concentrated and regular energy points. The difference is also consistent with the human eye's intuitive perception of the stylistic characteristics of realistic and anime images; i.e., natural photos are more colorful and detailed. In contrast, anime images have clear borders, more color mutations, and block-like distribution.

The spectrogram of an image does not have the semantic information and spatial coordinate correspondence of the original photo but more reflects the color distribution and changes in the picture. When using unpaired data to extract the image domain styles, the spectrogram analysis removes the redundant semantic information, enabling the discriminator to better focus on the style information of the image and learn the potential style distribution and the mapping relationship between the two domains. Thus, this paper proposes a style loss function based on the difference in spectral features *L*_frequency_. *X* represents the actual domain image, *Y* represents the reference anime domain image, *G* is the generator network, *D* is the discriminator network, and *F*_*dft*_ is the two-dimensional Fourier transform.

(4) $$\begin{array}{c} L_{\text{frequency}}=\log\;D\left(F_{dft}\left(y\right)\right)-E_{y}. \end{array}$$

The image animation platform aims to provide users with a convenient and efficient interface to convert images and videos to animation through simple page interactions. From the engineering design perspective, the platform system is divided into three parts: web front-end, system function, and core dependency. The web front-end consists of page display and user interaction, which allow users to interact with the server and display data. The system functions are mainly logic control, user management, and image generation. The business logic platform module realizes user management, the algorithm platform module recognizes image generation, and logic interaction is involved in both modules to control data flow and exchange. The platform comprises three main functions: front-end interface interaction, server logic processing, model generation, and video processing. The details are as follows.

1. The user submits the image or video to be converted through the front-end display interface.
2. The data is sent to the server over the network, and the service implemented by the Akka framework responds to it.
3. The business logic platform sends data information and transformation requests to the algorithm platform side.
4. After the algorithm platform completes the data transformation, it sends the data-related information to the business logic platform.
5. The business logic platform sends the converted images and videos to the user site through the network.

For the user interaction module and responding to front-end requests, the business logic platform needs to confirm and distinguish user identities to ensure that no data is transmitted incorrectly in the case of multiple users. On the other hand, the model interaction module is used for resource location information communication and message notification. The parameter metrics of the network model are shown in Figure 4. The Akka framework of the business logic platform uses the Actor model for thread interaction control. Each Actor can be regarded as an abstracted lightweight entity thread to control and process the program. The Actor has a management mechanism; i.e., the parent Actor can generate child Actors. The child Actors' survival cycle and related information are managed by the parent Actor [26]. In this system process, after the user sends a request, it is received by the Actor Manager, which generates a child Actor with unique ID identification according to the user information binding. It informs the child Actor of the content of this user's request. This child Actor processes the subsequent model platform interaction and user data transmission to ensure data flow. There are two functions for the algorithm platform module: one is to execute the animation conversion algorithm on the input image, and the other is to perform frame splitting processing and group frame reconstruction on the input video. When the input is an image, it is sent to the corresponding network for an animation image generation according to the model selected by the user. When the information is video, the video is firstly split into image frames and then sent to the corresponding network for batch conversion. Then, the images are composed into video in order frame by frame. This is the overall design architecture and implementation principle of the image animation platform system.

## 5. Analysis of Results

### 5.1. Deep Neural Network Model Analysis

Aiming at the characteristics of anime creation itself, the convolutional neural network structure is improved. The multilayer aggregation rescaled sentiment feature optimization module is proposed to enhance sentiment features in the middle layer and strengthen the elements that contribute a lot to the classification results and suppress the features that have a weak sentiment relationship with anime-style to improve the recognition ability of the network. Most of the recent literature uses CNN to extract features. Most of the existing literature analyzes them for the deep layer features of the network. In contrast, the process of CNN feature propagation to the deep layer inevitably loses some shallow simple features such as lines and textures due to pooling and other operations, which do not meet the needs of anime creation psychological feature extraction. As the brush lines of animation creation are the primary expression form of painter's psychology, the brush lines will show various textures under different painting techniques and different emotion-driven, which is a style feature of animation creation that cannot be ignored. For example, if the lines are straight and strong, neat, and straightforward, the painter's open-mindedness and solid and proud attitude will be between the brush and ink while the smooth and light, continuous and winding, steady and rhythmic lines will show the beauty of harmony and tranquility. Therefore, the existing algorithm cannot be used directly to obtain the action style characteristics. In this chapter, we improve the internal structure of the Res Net-50 convolutional neural network and propose a multilayer aggregated rescaled sentiment feature module based on the advantages of its constant mapping [27]. The module constructs a multilayer aggregated feature rescaling structure based on the residual module, implements multiple convolutional layer feature information aggregations in one module, feeds the aggregated information to the convolutional layer output, rescales the activation strength of the module unit for different features, and improves the network structure of the convolutional neural network to highlight the feature activation responses related to the emotional information of Chinese paintings and improve the network's ability to recognize the emotion of Chinese paintings. The structure of the proposed feature rescaling module for deep aggregation is shown in Figure 5. *X* represents the input, *Y* represents the output, and different colors are used to label other vectors or channel dimensions. The green module output dimension is *d*, the blue output dimension is *c*, and the orange output dimension is *c*/*∂*. The design structure can share the features of CNN multilayer convolutional layers, which can take advantage of the deep layer network to extract *X Yc* features with more actual semantic meaning and more global, i.e., the abstract emotional information presented in composition, the overall atmosphere, etc. It can also obtain the features of the external layer network to extract simple local information. While getting the overall emotional mood of Chinese painting, it considers the local details such as points and lines to express emotion.

Let the dimension of input *X* be *h* × *b* × *c*, and the output of the 1st convolutional layer is *A*^1^, then, *A*_1_=*w*_1_ ⊗ *X*, where ⊗ is the convolution operation, and *w*_1_ is the kernel parameter. The bias term is ignored in the Equation for expressive clarity and simplicity. The *h* × *b* × *c*-dimensional convolutional layer output *A* is compressed by global average pooling into vector *g*(*A*), which means the global features represented by each channel are counted separately. The *k*th element of the vector *g*(*A*) is denoted as

(5) $$\begin{array}{c} g\left(A\right)=\sum_{i}A_{ij}^{k}-\frac{h-1}{\sqrt{h\times b\times c}}, \end{array}$$

where *A*_*ij*_^*k*^ are the *kt*h channel row and column elements of the convolutional layer *A*. The vectors after the global average pooling operation of the three convolutional layers in the module are obtained from the above equation and expressed as *g*(*A*1), *g*(*A*2), and *g*(*A*3), respectively. The elements in the vector represent the feature information of each channel of the corresponding convolutional layer. The feature scale of information representation depends on the depth of the convolutional layer: the shallow layer of the network, due to the large resolution of the input or feature map, the convolutional kernel learns small-scale information such as points, lines, and textures, and then the corresponding convolutional layer channels represent the local detail features in the image; the deep layer of the network, due to the small resolution of the feature map, the convolutional kernel learns large-scale information, and the corresponding convolutional layer channels represent the overall abstract features of the image such as depicted objects and emotional atmosphere. *gk*(*A*) statistically calculates the activation of an element in the *k*th channel of convolutional layer *A* in the global range of the image. Due to the bottleneck structure of the residual module, vectors *g*(*A*1) and *g*(*A*2) of dimension *d* and *g*(*A*3) of dimension *c*, i.e., corresponding to the number of channels of the corresponding convolutional layer (*d* < *c*), cannot be aggregated directly. Therefore, *g*(*A*1) and *g*(*A*2) with the same dimension are aggregated. Then, the vector dimension is raised to the *c* dimension through the fully connected layer and then aggregated with *g*(*A*3), and the resulting vector *e* is calculated as follows:

(6) $$\begin{array}{c} e=\sum_{\partial =1}\frac{g\left(A3\right)}{g\left(A1\right)+g\left(A2\right)}-1. \end{array}$$

Next, the weight vectors *l*: *l*=*∂*(*w*_3_*δ*(*w*_2_*e*)) are trained using two fully connected layers, where *w*_2_ ∈ *c*/*δ* × *cw*_3_ ∈ *c* × *c*/*δw*_2_ are the descending layer's parameters and the ascending layer's parameters, i.e., the two fully connected layers, form the bottleneck structure. The two fully connected layers are set with the adaptive activation function and activation function defined in the equation, respectively, which mainly serve to enrich the nonlinear transformation of the network and enhance the channel feature importance extraction ability of the aggregation module. In contrast, the Sigmoid activation function mainly serves to increase the nonlinear elements but also normalize the input to *lk* and is the *k* aspect of the c-dimensional vector *l*, which indicates the global feature activation size of the *k* channel. The bottleneck structure of dimensionality reduction followed by dimensionality increase reduces the network complexity and prevents overfitting, on the one hand, and dramatically reduces the number of training parameters and computational effort, on the other hand, according to the actual training effect, where/is the dimensional change ratio. Finally, the weights *l* are used to rescale each channel feature of *A*_3_ and set *y*_*k*_ as the mapping of the *k* channel of the module output *y*.

(7) $$\begin{array}{c} y_{k}=\int \frac{l_{k}}{\sqrt{A_{3k}-x_{k}}}. \end{array}$$

*A*_3*k*_ and *xk* denote the 3rd channel mapping of the *k* layer convolution output and the *k* input channel mapping *x*, respectively; the *l* vector elements are trained to express the importance of the corresponding *A*_3_ channel features for obtaining the emotional information of Chinese paintings. The channel features output by the rescaling module enhances the feature responses that are closely related to the dynamic classification and suppresses the feature responses that have little relationship with the emotion of Chinese paintings, to obtain better emotional features. The proposed multilayer aggregated feature rescaling module is used to connect to form the overall network, and the network loss function is expressed as

(8) $$\begin{array}{c} L=\sum_{i}\frac{1}{U}-\sum_{m}p_{i}-\frac{\log\;p^{m}}{p_{i}}. \end{array}$$

### 5.2. Painter Psychology and Animation Creation Style Realization

The natural way to extend image processing techniques to video is to execute images frame by frame and then concatenate each frame to encapsulate them into a video. However, this scheme may introduce temporal inconsistencies, leading to flicker and jitter in the video. In the style migration task, the style and content of the images are split, and the style representation of the style image is combined with the content image to generate a stylized image. When extending this work to video style migration, although the difference in semantic information between frames is slight, the difference in the stylized pictures is significant. This difference comes from the inherent instability of the GramMatrix method, which allows small local changes to have a relatively significant impact overall.

For this reason, some studies have used optical flow methods to constrain this temporal consistency *P*, 36.2% by controlling the generation of subsequent frames through the visual flow information and masking the performance of the preceding structures. Instability also arises in image translation tasks such as coloring and segmentation when extended to video. This instability stems from the excessive difference between the two domains, where the image has more generative space and “creativity” during the transformation [28]. Therefore, small changes in the source image may cause significant fluctuations and effects on the conversion of the whole idea. Vide02Vide04 controls the image conversion between consecutive frames to reduce jitter by introducing optical flow information and reinforcing constraints by modeling the foreground and background separately. The video conversion results are shown in Figure 6.

To demonstrate the effectiveness of the proposed multilayer feature aggregation rescaling module, this chapter compresses the classification results of the network before and after rescaling. The Res Net-50 network structure is divided into four stages according to the output size of the convolutional layer. Stages 1 to 4 from the input to the output comprise 3, 4, 6, and 8 residual modules. Since deeper features directly impact the classification results, this chapter optimizes the residual modules from stage 4 to stage 1 of the network into the proposed feature aggregation rescaling modules, starting from the deeper layers. The number of optimized modules is 16, which means the optimized network structure in this chapter. From the experimental results, it can be obtained that the accuracy of emotion classification gradually increases with the increase of the number of optimization modules, which indicates that the proposed multilayer feature aggregation rescaling module effectively improves the features extracted by the network and has a significant improvement on the model performance, which is beneficial to the recognition of the psychology of anime creation painters. The optimization effect of the feature aggregation rescaling module is shown in Figure 7.

This paper analyzes the interframe images when extending scene image animation to the video domain. In most cases, the videos can maintain their original stability better and do not show more considerable jitter than the style mentioned above for migration and image translation tasks. This section uses FSGAN and AFGAN to animate and transform the video images, respectively, and they are extracted frame by frame for comparison and analysis. For the convenience of exposition, only one image is removed from the video every three frames interval here, and four frames are extracted for analysis. (a) is the original video image frame, and (b) is the FSGAN converted video image frame. FSGAN network maintains the semantics of the original image better, so the slight differences between structures do not cause the interframe jitter problem. AFGAN, although the abstracted color blocks and edge lines are more pronounced, this change depends on the overall pixel distribution and characteristics and the impact of the slight differences between frames on the local structure. The effect of subtle differences between frames on the local network does not expand in the conversion. The appearance of color blocks and edge lines can be stable from the conversion results. The information retention of the original image is much higher for the animation than for other conversion tasks, and the source image is more constrained to the generated image. And its style of conversion is almost mapped based on the pixel level, and the change of local position does not impact other regions. The generator uses bilinear interpolation and nearest-neighbor interpolation algorithms in the upsampling process. The pixel-to-pixel expansion is more stable when combined with adequate preservation of the original image information. Therefore, the generated results of the image network can be directly extended to the video task for video animation. It should be noted that the research of AFGAN is mainly used for portrait animation, in which there are specific requirements for face occupancy and face orientation so that instability will occur for continuous frame images with significant changes in face regions. However, AFGAN can still maintain good temporal stability when acting on videos with a pure background. Its animation style is more abstract and depends on the overall tone of the training portrait set compared to FSGAN. A comparison of the results before and after video conversion is shown in Figure 8.

## 6. Conclusion

In this paper, we study the essential components of a convolutional neural network and its working principle, and based on the understanding and mastery, we propose the dual-core compressed activation module (DSKE) to extract the overall features and local detail features of anime creation according to the working principle between network modules and the characteristics between anime creation styles. The anime styles are processed for data enhancement; Then, the convolutional neural network is built with the DKSE module and several depth-separable convolutions to realize the effective classification of anime creation styles. The experimental validation of the anime-style classification algorithm based on the dual-core compressed activation neural network proposed in this paper is carried out. The experimental validation results show that the data enhancement process of the samples can effectively improve the classification accuracy; the effect of the parameters of the dual-core compressed activation module on the classification of the model is verified, and a good set of module configuration parameters is obtained; the Grad-CAM algorithm is used to visualize and analyze the regions that the network model depends on during the learning process, and the analysis results show that the network of this paper can better extract the overall features of the images. The analysis results show that the web in this paper extracts the general characteristics and local detail features of the image well; this paper proposes a deep network feature aggregation rescaling algorithm for the mental classification of anime creation. The global information of the features of each convolutional layer within the aggregated network module is used to make full use of the pencil line features extracted from the shallow layer of the network and the advanced emotional semantic features in the deep layer. Finally, the obtained information is used to recalibrate the output features to get parts with more profitable relationships between painterly psychology and anime creation style.

## Figures and Tables

**Figure 1:** Le Net network structure.

**Figure 2:** Example of pooling layer.

**Figure 3:** Comparison of spectrum features in realistic domain and animation domain.

**Figure 4:** Parameter indicators of the network model.

**Figure 5:** Feature recalibration module for multilayer aggregation.

**Figure 6:** Video conversion results.

**Figure 7:** Optimization effect of feature aggregation recalibration module.

**Figure 8:** Comparison of results before and after video conversion.

## Data Availability

The data used to support the findings of this study are included within the article.
